RETRACTED

# Application of Data Mining in the Effect of Traditional Chinese Medicine on the Rehabilitation of Cerebral Spasticity of Lower Extremity Exercise Energy

**DOI:** 10.1155/2022/9746906

**Published:** 2022-02-18

**Authors:** Jing Du, Yiran Liu

**Affiliations:** ^1^Rehabilitation Department of Traditional Chinese Medicine, Hanyang Hospital of Wuhan University of Science and Technology, Wuhan 430000, China; ^2^Hubei Provincial Hospital of Traditional Chinese Medicine, Wuhan 430000, China

## Abstract

In this article, we have examined the effect of acupoint injection of mecobalamin on the nerve function of the lower limbs of stroke patients by giving acupoint injection of mecobalamin for 2 weeks in patients with stroke, effectively fusing acupuncture, acupoints, and drugs in traditional Chinese medicine to rehabilitate the effect of motor function and activities of daily living. For this purpose, a total of 60 study cases will be screened in the study. They are randomly divided into experimental group and control group: the control group will be treated with conventional stroke treatment and nursing, and the experimental group will be treated with bilateral acupoint injection of mecobalamin; once a day, after 14 days of continuous injection, we observed and intervened the lower limb nerve function, motor function, and activities of daily living of the two groups before and after the treatment and statistically analyzed the data so as to obtain the clinical effect of the treatment on the lower limb rehabilitation of stroke patients. Before the intervention, the general information and basic clinical data of the two groups of subjects were collected for baseline comparison, and the differences between the two groups of subjects' lower limb nerve function, motor function and activities of daily living before the intervention were compared. Comparison of lower limb neurological deficits mainly include comparison between groups and comparison within groups. Comparison of lower limb motor function mainly include comparison between groups and comparison within groups. (1) Acupoint injection of mecobalamin therapy and simple stroke rehabilitation therapy have good results. (2) Acupoint injection of mecobalamin can improve the neurological deficits of the lower limbs of stroke patients more than simple conventional stroke therapy, and it also has a rehabilitation effect in nourishing the nerves, improving circulation, and protecting the brain. (3) Point-injection mecobalamin therapy is more effective than conventional stroke therapy in improving the motor function of the lower limbs and promoting the rehabilitation of the lower limbs of patients with ischemic stroke. (4) Acupoint injection of mecobalamin therapy can improve the activities of daily living of patients with ischemic stroke and improve the quality of life of patients compared with conventional stroke therapy alone.

RETRACTED

## 1. Introduction

Stroke is a very common type of disease among cerebrovascular diseases today. It is also a chronic non-communicable disease recognized by the world as extremely dangerous [1]. It is called apoplexy or stroke in Chinese medicine. In China, the number of cerebrovascular diseases has reached 7 million people, of which ischemic stroke accounts for more than 80% [2]. The incidence is 120–180/100,000, and the fatality rate is 60–120/100,000. The disability rate reaches 75% [3]. In our country, although the continued economic prosperity and development has brought about the double improvement of material and spiritual conditions, some people have not developed good dining habits and regular work and rest habits. In addition to the increase in the elderly over 60 years old, people suffer from stroke. The number of people has shown an upward trend year by year, among which the number of ischemic stroke occurrences has increased the most [4]. The disease shows a trend of rejuvenation, disability, and damage rates. In addition, its incidence is also closely related to genetic and environmental effects, which seriously endangers the health of people of different ages, races, and regions [5]. Stroke patients often have sequelae such as increased muscle tone, muscle spasm, pain, joint contractures, and so on within one month after the first onset, especially muscle spasm, which causes the limbs to be unable to move normally, and the patient's self-care ability is impaired to work, study, and so on. Life is dependent on medical staff or relatives and friends, and the quality of life has plummeted.

Therefore, as soon as possible, research and discuss more scientific, effective, simple, and easy intervention and rehabilitation measures to effectively relieve the spasm of the limbs of stroke patients so that they can recover their body and mind as soon as possible, and it is urgent to return to the family and society. Traditional Chinese medicine believes that stroke is caused by cerebral arterial obstruction and wind evil invades the body. The patient's limb hemorrhage failure is the result of poor blood circulation, qi deficiency and blood stasis, and loss of nourishment. There are many clinical therapies to treat stroke, and they are becoming more diversified. Acupuncture (as shown in Figure 1), physiotherapy, surgery, and other therapies have their own magical powers. Although they all have certain effects, their curative effects are also mixed. Their application and promotion are often affected by factors such as the level of medical care, medical expenses, equipment technology, and patient tolerance. In recent years, among many stroke diagnosis and treatment programs, the combined therapy of Chinese and Western medicine has sprung up, especially the acupoint injection method. This method not only inherits the traditional Chinese medicine syndrome differentiation and treatment, the theory of meridians, and the essence of acupuncture but also retains the western medicine injection therapy. The advantages of acupuncture, acupoints, and medication are combined into one. In clinical practice, it has been found that the rehabilitation application of acupoint injection for the treatment of stroke and its sequelae is more and more extensive, especially for the treatment of hemiplegia after stroke. Acupoint injection, as an extended technique of traditional Chinese acupuncture and a modern new type of therapy, has gradually revealed its advantages.

RETRACTED

In this article, we have examined the effect of acupoint injection of mecobalamin on the nerve function of the lower limbs of stroke patients by giving acupoint injection of mecobalamin for 2 weeks in patients with stroke, effectively fusing acupuncture, acupoints, and drugs in traditional Chinese medicine to rehabilitate the effect of motor function and activities of daily living. For this purpose, a total of 60 study cases will be screened in the study. They are randomly divided into experimental group and control group; the control group will be treated with conventional stroke treatment and nursing, and the experimental group will be treated with bilateral acupoint injection of mecobalamin; once a day, after 14 days of continuous injection, we observed the lower limb nerve function, motor function, and activities of daily living of the two groups before and after the intervention and statistically analyzed the data to obtain the clinical effect of this therapy on the lower limb rehabilitation of stroke patients.

The rest of the manuscript is organized according to the following agenda items.

In Section 2, a comprehensive review of the existing state-of-the-art mechanism, which is published in well-reputed journals and conferences, is provided along with various issues in these schemes. Then, in the subsequent section, material and methods were presented with sufficient detailed information. In Section 4, experimental results and observations were described in detail that is followed by comprehensive concluding remarks and future directives.

## 2. Related Work

At present, in the prevention and treatment of cerebrovascular disease, there is no immediate and very reliable treatment and effect at home and abroad. Therefore, actively exploring the risk factors of stroke can provide reliable evidence for clinical and guide the prevention and treatment of stroke to be more scientific and effective. Standardized and effective development; (1) Western medicine's understanding of stroke: Western medicine generally believes that stroke is not the outcome of a single factor. Blood pressure, blood sugar, and hyperlipidemia are all factors that cause damage to stroke. Older people, atrial fibrillation, and transient ischemic attack (TIA) are also high-risk groups. Risk factors such as high homocysteine (Hey), high C-reactive protein (CRP), inflammatory response, high fibrinogen, and metabolic syndrome have also been explored day by day, attracting public attention. Sun and others concluded that in addition to the above factors, there are also metabolic syndrome and gout. In summary, stroke patients usually suffer from multiple causes. (2) TCM's understanding of stroke: TCM also believes that the cause of stroke is not the result of a single factor. Stroke can be caused by the invasion of wind (such as liver wind and external wind). Rising due to fire (such as liver fire and heart fire) can also cause stroke. If the patient is trapped by wind and damp phlegm, stroke can also be induced. People with yin and qi deficiencies have a high probability of stroke. People who are chronically ill and have unclear internal toxins are also prone to stroke. In addition, emotions can also affect human health, and those who are overwhelmed or worried about grief can also easily cause stroke. When the climate changes, sudden cold will invade cold pathogens, poor circulation, poor circulation of qi and blood, stasis caused by qi deficiency, and stagnation of essence and qi that are all incentives.

RETRACTED

The motherland's TCM is extensive and profound, and TCM has its unique advantages in the treatment of stroke. It is based on the theory of “yin and yang and five elements”; with “syndrome differentiation and treatment” as the main principle, focusing on “seeing, hearing, asking and cutting” to comprehensively collect data on stroke patients; focusing on the analysis and discussion of etiology, disease, location, and pathogenesis; and observing the internal organs, meridians and collaterals of the human body, joints, qi and blood, and so on infer the relationship between the evil and the positive and the ebb and flow, summarize the syndrome types, and use this to implement targeted therapies. Acupuncture therapy, also known as acupuncture or acupuncture, is a unique medical method of traditional Chinese medicine. It is based on the theory of traditional Chinese medicine. It uses different needles to penetrate the face points and stimulate the meridians to prevent and treat diseases. Among them, acupoint injection is one of the important treatment and nursing techniques in traditional Chinese medicine. In the old days, it was also called the “face injection method” or “water acupuncture method.” The therapy is based on syndrome differentiation and meridian theory to cure diseases. Through the injection of a small dose of the medicinal solution to the acupoints, the three effects of acupuncture, pharmacology, and acupoints are effectively integrated. This method was first started in the 1950s as the “golden needle” of acupuncture and moxibustion, and it has advanced with the times. In clinical application, the golden needle was replaced by a syringe, and the advantages and essence of traditional Chinese acupuncture therapy and western medicine injection therapy have been continuously absorbed, and acupuncture has been fully utilized. The multiple effects of meridians, acupoints, and drugs eventually evolved into a more complete theory, higher technological content, better curative effect, wider application, and promising therapy.

In recent years, there have been many studies on the treatment of limb spasm after stroke. Acupuncture alone, acupuncture combined with electroacupuncture, scalp acupuncture, Jiaji points, drugs, rehabilitation, and so on have achieved certain effects and are positive for functional reconstruction after brain injury. In terms of therapeutic function, acupuncture and moxibustion are important methods to treat hemiplegic limb spasm after stroke. Lee [6] combined the neuroanatomy of modern medicine with the meridian points of traditional medicine and took acupuncture to antagonize the muscle group points to treat stroke. Zhang et al. [7] used acupuncture to coordinate muscle tension balance to treat stroke spastic paralysis. Pan [8] used penetration acupuncture and electric acupuncture to treat increased muscle tension after stroke. In Liu and Miao's [9] study, the effect of electro-acupuncture combined with rehabilitation therapy on muscle spasm after stroke was treated with electro-acupuncture combined with rehabilitation therapy. Wang and Liu [10] used Tongluo Shujin Liniment plus massage to treat increased muscle tone after stroke, but it is not yet found that there are documents discussing its long-term functional indicators, lack of long-term follow-up for more than one month, and few reports of adverse reactions, only studying this process during hospitalization, so it suggests that in future, TCM efficacy research should be more rigorous and standardized clinical trials. Design and persuasiveness can improve the reliability of conclusions.

RETRACTED

## 3. Proposed Methodology

### 3.1. Sample Size Estimation

Let us refer to the sample size estimation formula in Hu l PS Medical Statistics Manual:

(1) $$\begin{array}{c} n=\pi_{0}\left(1-\pi_{0}\right)\frac{\left(U_{2\alpha }+U_{2\beta }\right)}{\delta^{2}}, \end{array}$$

where *δ*=(*π* − *π*_0_), *π* is the effective rate of the test group, and *π*_0_ is the effective rate of the control group. According to *α*=0.05, *β*=0.1, *U*_2*α*_=1.645 (one-sided), *U*_2*β*_=1.282, refer to related literature *π* is 93.3%, and *π*_0_ is 66.7%. Put the above data into the formula to get out of *n* ≈ 26.89. Taking into account the loss to follow-up rate of 10%, each group needs to include 30 cases.

### 3.2. Research Methods

Cases that meet the requirements are numbered according to the order in which they entered the study. Look up the random number table to generate a random sequence. Randomization is divided into A (experimental) group and B (control) group. There were 30 cases in each group. In the intervention program, the control group received conventional treatment and nursing care (30 cases), and the test group received acupoint injection therapy (30 cases) on this basis. All patients received routine treatment and care for stroke. Routine care includes psychological care, food care, respiratory care, limb care, and exercise.

#### 3.2.1. Acupoint Injection Therapy

1. Pretest preparation: before the intervention, train the nursing staff of the test group patients who performed acupoint injections during the hospitalization period, including the positioning of acupoints, acupuncture techniques, precautions, and so on. After the training, the assessment was carried out, and both assessments were qualified (both ≥80 points) can enter the formal test
2. Point selection: choose Zusanli points on both sides.
3. Positioning: anterolateral calf 3 inches below the calf nose and a transverse finger in front of the tibia.
4. Drug selection: methazolamide injection is used.
5. Needle selection: disposable sterile syringe 2.5 ml with a needle.
6. Specific operations.

#### 3.2.2. Evaluation Index

General index: (1) basic indicators: (recorded once at the time of enrollment) on the day of enrollment, collect the general information of the two groups of subjects. Mainly include name, gender, age, marriage status, education level occupation, and so on. The basic clinical information involves medical history medication comorbidities and so on and (2) adverse events: Adverse events should be prevented first, and emergency plans should be prepared. If adverse events occur, they should be recorded and reported in time, including start and end time duration emergency treatment prognosis and so on. Record the occurrence time, duration, end time, characteristics, corresponding treatment measures, and outcome of adverse events at any time.

RETRACTED

Efficacy index:

1. Neurological function: the National Institutes of Health Stroke Scale (NIHSS) scale is a kind of evaluation scale that is widely used in clinical practice and is time-saving and convenient. It is a table specifically for neurological function assessment. Different types of stroke can be assessed by this table. Its content is more comprehensive, with high reliability and validity. The reliability of internal consistency is better. Su [11] has already explained this in the literature. Wang et al. [12] researched that the NIHSS scale contains vertebrobasilar system stroke examination items, which have high inter-rater reliability, test-retest reliability, and validity. The neurological deficit assessment scale (lower extremity) used in this study has 2 main contents. In order to evaluate lower limb muscle strength and walking ability, we set the highest score and the lowest score. The highest score is 12 points, and the lowest can be 0 points. The higher the score, the more serious the neurological deficit.
2. Motor function: the simplified FMA motor function assessment scale (lower limbs) includes 7 major items, with a total score of 34 points. It is subdivided into 17 subitems, each with a minimum of 0 points and a maximum of 2 points. The lower the score, the worse the lower limb motor function, and vice versa. The simplified FMA motor function assessment scale is divided into upper and lower limbs. According to the focus of this research, the simplified FMA motor function scale (lower extremity; FMA) is selected to evaluate the motor function of the lower limbs of stroke patients. It assesses seven aspects of the patient's lying position, sitting position, and standing position. There are multiple research items related to limb reflex, cooperative movement, ability, speed, and so on. Each item is subdivided into 3 grades, with the lowest grade being 0 points and the highest being 2 points. The highest score for the lower limbs in this table is 34 points. The lower the score, the worse the movement of the lower limbs. On the contrary, the higher the score, the better the motor function.
3. Activities of daily living: Modified Barth index (MBI) rating scale (lower limbs) is used. The full score of the MBI scale is 45 points. The higher the score, the better the patient can take care of himself. Conversely, the lower the score, the heavier the dependence on caregivers. Its predecessor is Barthel index (BI), which is an assessment of the prognosis of acute stroke. It is widely used all over the world, with good reliability and validity.

RETRACTED

### 3.3. Data Processing and Methods

#### 3.3.1. Evaluation Standards

Record each time before and after the intervention and observe the changes in the following three indicators and scoring before and after the intervention.

1. Several prognostic lower limb neurological deficits NIHSS scores decreased, and there were statistical differences (*P* < 0.05), indicating that intervention is meaningful.
2. The FMA score of lower limb motor function in several prognoses is improved, and there is a statistical difference (*P* < 0.05), which indicates that the intervention is meaningful.
3. The MBI scores of the lower extremity activities of daily living have improved in some prognoses, and there are statistical differences (*P* < 0.05), indicating that the intervention is meaningful.

#### 3.3.2. Data Processing

All statistical analysis in this study was processed with SPSS 18.0 statistical software package. To ensure that the data is accurate and not biased, it is entered by two persons. First, enter the collected data into the Excel table and then import it into the SPSS 18.0 software to perform statistical analysis of the data.

1. Measurement data: the normal distribution is represented by $\bar{x}\pm s$. For comparison between groups, the data satisfy normality, and the independent sample test is not satisfied using the rank-sum test. In comparison between the two groups, the difference satisfies normality, using a paired *t* test. The unsatisfied ones use the rank-sum test.
2. Counting data: it can be expressed by frequency (*f*), composition ratio or percentage (*P*), and average rank $\left(\bar{R}\right)$. The counting data is tested by *x*^2^.
3. Grade data: the rank-sum test is used.
4. Inspection level: *α*=0.05; when *P* < 0.05, the difference is statistically significant.

(2) $$\begin{array}{c} \bar{x}=\frac{\sum_{i=1}^{n}x_{i}}{n}. \end{array}$$

#### 3.3.3. Data Comparison Method

General information comparison: (1) Two groups of gender, age, occupation, culture, hemiplegia: use chi-square test; (2) Two groups of disease course: satisfy normality and homogeneity of variance, select two independent samples and test; (3) The use of antihypertensive drugs in the two groups: the rank-sum test of grade data was selected. The two groups took drugs for activating blood circulation and collaterals and antiplatelet aggregation drugs: Chi-square test was used.

NIHSS score comparison:

1. Comparison between groups before intervention: To meet normality and homogeneity of variance, conduct two independent samples and test.
2. Intra-group comparison before and after intervention: The two groups were compared before and after the intervention in this group. Because the difference satisfies the test of normality and homogeneity of variance, the paired *t* test is used.
3. Comparison between groups after intervention: After the intervention, the two groups are scored because the values meet normality and homogeneity of variance. Two independent samples are selected and tested.

RETRACTED

FMA score comparison:

1. Comparison between groups before intervention: carry out two independent samples and test;
2. Intra-group comparison before and after intervention: the two groups were compared before and after the intervention in this group, respectively. Because the difference satisfies the test of normality and homogeneity of variance, matching and testing are selected.
3. Comparison between groups after intervention: carry out two independent samples, test, and analyze.

MBI index comparison:

1. Comparison between groups before intervention: compare the MBI scores of the two groups of patients before the intervention. Since the MBI index does not conform to the normal distribution, a non-parametric test was used to compare the MBI index between the two groups;
2. Intra-group comparison before and after intervention: the test group and the control group were compared before and after the intervention score comparison; the difference normality test is not satisfied; and the paired rank-sum test is selected;
3. Comparison between groups after intervention: after the intervention, the MBI scores of the two groups of patients were compared. Because the normality test was not satisfied, the rank-sum test of two independent samples was selected.

## 4. Experiments and Results

### 4.1. Test Completion

A total of 60 study cases were screened out in this study. These patients were diagnosed with ischemic stroke in the brain department (inpatient department) of a tertiary hospital. They were randomly divided into test group and control group (30 cases each). The control group received routine care for stroke. The experimental group added acupoint injection therapy on this basis. It was injected once a day, and there were no adverse events in the patient for 14 consecutive days during the entire trial. Because the Chinese medicine method is deeply rooted in the hearts of the people, the acupoint injection therapy is well taught; the doctors and nurses are professionally responsible; and the overall cooperation of the subjects is good. None of the study subjects had withdrawn or lost to follow up. The patient's compliance was high, and the trial was successfully completed.

RETRACTED

### 4.2. Baseline Analysis

1. Comparison of the age and course of disease between the two groups before the intervention: the age and disease course of the two groups of patients were collected, and two independent samples were used for i-test. The data show *P* < 0.05, which is not statistically significant. The two groups of patients had no difference in age and course of the disease, and they were comparable (see Table 1 for details).
2. Comparison of medication use between two groups of patients before intervention before the intervention: the two groups of patients taking antihypertensive drugs were tested by chi-square method, while those taking blood-activating and collateral drugs and antiplatelet aggregation drugs were tested by data rank-sum test. The difference was not statistically significant (*P* < 0.05) indicating that there is no difference in medication. There is no difference in medication (see Table 2 for details).
3. Comparison of the lower limb NIHSS score, FMA score, and MBI index of the two groups of patients before intervention: before the intervention, the NIHSS score and FMA score of the lower limbs of the two groups of patients were tested for homogeneity of variance, and the results showed homogeneity of variance (*F*=0.932, *P*=0.338; *F*=0.109, *P*=0.743), so the analysis/test was used to compare the results. This shows that there is no statistical difference between the groups (*P* < 0.05). Since the MBI index does not conform to a normal distribution, a non-parametric test is used. The difference in the following table is not statistically different (*P* < 0.05), indicating that there is no difference in the score between the two groups before the intervention, in comparison (see Tables 3, 4 for details).

### 4.3. Test Results

1. Comparison within the group: after the intervention, the lower extremity NIHSS score, FMA score, and MBI index scores of the experimental group and the control group were collected and compared within the group.
2. Control group: after the intervention, the lower limb NIHSS score of the patients decreased compared with the preintervention score, and the FMA score and MBI index scores were higher than those before the intervention, and the differences were statistically different (*P* < 0.05) (see Figures 2 and 3).
3. Test group: after the intervention, the NIHSS score, FMA score, and MBI index of the patients after the intervention were compared with those before the intervention. The NIHSS score of the lower limbs of the patients decreased compared with the scores before the intervention (see Figures 4 and 5 for details).
4. Comparison between groups: through the comparison between groups, the homogeneity of variance test was performed, and the results showed the homogeneity of variance (*F*=2.403, *P*=0.134; *F*=0.127, *P*=0.723), Therefore, two independent sample (*t*) tests are used for analysis and comparison. The results showed that the NIHSS score of lower limb neurological deficits of the experimental group was lower than that of the control group after intervention, and there was a statistical difference (*P* < 0.05), indicating that the intervention was meaningful (see Figure 5 for details). Through the comparison between the groups, the FMA score of lower limb motor function of the experimental group was higher than that of the control group after the intervention, and there was a statistical difference (*P* < 0.05), indicating that the intervention was meaningful (see Figure 6 for details). Through the comparison between the groups, the MBI scores of the patients in the test group were higher than those in the control group after the intervention, and there was a statistical difference (*P* < 0.05), indicating that the intervention was meaningful (see Figure 7 for details).

RETRACTED

### 4.4. Discussion

Comprehensive and systematic evaluation through multiangle, multidirectional, and correspondingly complementary scales can more scientifically, systematically, and intuitively evaluate the actual effect of the implemented acupoint injection intervention measures on the rehabilitation of the lower extremity function of stroke patients.

#### 4.4.1. The Effect of Injection of Methazolamide on the Neurological Deficits

In terms of neurological evaluation of stroke, the National Institutes of Health Stroke Scale (NIHSS) is a stroke evaluation scale that is widely used clinically, saves time, is convenient, has high reliability and validity, and has a more comprehensive content. It is suitable for various types of strokes, especially for the assessment of neurological deficits in the acute phase of stroke and strokes in the cervical and vertebrobasilar arteries. It is often used by physicians to evaluate disease outcomes and prognoses [13]. From the results of the research data, it can be seen that the use of methazolamide injection at acupoints does have a certain improvement effect on patients' neurological deficits. The principle and mechanism are analyzed as follows: (1) acupoint injection can stimulate nerves and stimulate body fluid regulation. Acupoint injection is to use a syringe needle to aspirate medicinal liquid preparations and perform acupuncture on the corresponding acupoints of the patient's limbs. When the needle pierces the acupoints of the lower limbs, it immediately stimulates the abundant nerve-ending receptors in the lower limbs, triggering the generation and uploading of nerve impulses. To the advanced center, it stimulates the function of the hypothalamus-pituitary system and promotes more sensitive neurohumoral regulation [14]. (2) Acupoint injection can promote blood circulation and dredge collaterals and relieve pain. (3) Acupoint injection can nourish the nerves and promote the rehabilitation of lower limbs dominated by the nerves. (4) Acupoint injection can improve brain microcirculation and improve ischemia. The changes in cerebral microcirculation are achieved through a series of changes in hemorheology [15]. Acupuncture allows blood vessels to be expanded; resistance is reduced; and collateral branches are remodeled, so cerebral ischemia is naturally relieved and improved [16]. The activity of superoxide disproportionation is activated, which accelerates the elimination of free radicals [17] and makes cells more vigorous. Acupuncture can promote the nerve survival ability of the injured site [18] and promote neuron regeneration [19]. (5) The acupoint selected in this study is Zusanli, which is called a “healthy and longevity acupoint.” Stimulating this acupoint can strengthen the physique. To a certain extent, it improves the ability of stroke patients to resist disease. (6) The methazolamide injection for acupoint injection has a neuroprotective effect on its own curative effect. Its composition is an endogenous coenzyme B12, which is combined with glutathione to have defensive and therapeutic effects on neurotoxic reactions [20]. From the clinical research data in the table, it can be seen that the scores of the neurological deficit NIHSS (lower limbs) of stroke patients after the intervention are all lower than before the intervention, and there is a statistical difference (*P* < 0.05), which is statistically significant. Studies have shown that the effect of combined therapy with acupoint injection of methylazuramine is better than that of simple rehabilitation treatment, and the rehabilitation effect on lower limbs is also more obvious. The intervention measures of acupoint injection have more significance and advantages.

RETRACTED

#### 4.4.2. Effect of Acupoint Injection of Methazuramide on Motor Function

Studies have shown that the simplified FMA scale is objective, economical, simple, and convenient and is very suitable for the assessment of early stroke patients. It is currently recognized as an excellent assessment tool with good reliability and validity [21]. According to the focus of this research, the simplified FMA motor function scale (lower extremity; FMA) was selected to evaluate the lower extremity motor function of stroke patients. It assesses the patient's three postures in the supine position, the end sitting position, and the standing position, a total of seven aspects. It is to be checked whether the lower limbs have reflex activities, flexor coordinated movement, extensor coordinated movement, activities accompanied by coordinated movement, activities that depart from coordinated movement, normal reflex activities, coordination ability, and speed. There are a total of 17 aspects, each with 3 levels, each with a score of 0, 1, 2,…. The score for the lower limbs can be up to 34 points. The higher the score, the better the separation of the lower limbs. The motor function is affected. The degree of damage is less. The mechanism of acupoint injection to promote the rehabilitation of lower limb function of stroke patients is as follows: (1) acupoint injection can dredge the meridians and reconcile the balance of yin and yang. Acupoint injection can regulate qi and blood and nourish the limbs. Combined with the efficacy of the injected methazolamide drug itself, it can nourish nerves, nourish muscles and muscles, effectively improve peripheral neuropathy, reduce the level of homocysteine in patients with stroke, and reduce high-risk factors for stroke, so as to be effective in improving the patient's sensation, and mobility is conducive to the recovery of lower limb function. (2) Acupoint injection can also inhibit muscle spasm, promote joint mobility, and prevent limb disuse. (3) Zusanli can have an effect on the sense of movement and perception of the limbs. This is related to stimulating the specific brain area activated by the acupoint. It is generally believed that the central anterior gyrus may be related to the body motor function [22]. The central posterior gyrus is related to the sensory center of the body [23]. (4) Injecting methylazuramine during acupoint injection not only can stimulate the acupoints but also can have the effect of dredging the meridian qi and blood, relieving pain, and nourishing nerves. As a medicine that nourishes the nerves, methazolamide can effectively treat peripheral neuropathy. The drug can improve muscle weakness and muscle atrophy of the lower limbs and improve tendon reflexes and perception; it can prevent axon degeneration, repair damaged nerve tissue, and improve the function of the limbs innervated by the corresponding nerves. Research data shows that FMA (lower extremity) scores of stroke patients after intervention are all higher than before intervention, and there is a statistical difference (*P* < 0.05). The lower limb motor ability scores of the experimental group were higher than those of the control group, which was statistically significant, indicating that the intervention measures of acupoint injection are meaningful and have more advantages.

RETRACTED

#### 4.4.3. Effect of Acupoint Injection on Activities of Daily Living in Patients

The Bhattacharyya index (BI) is a widely used scale. It is a disability scale for the evaluation of prognosis and rehabilitation in the acute phase of stroke, but the scale is not enough to reflect the cognitive communication ability of patients. In this study, acupoint injection of methylazuramine combined with Zusanli point was used, and the dual effects of medicine points were used. On the one hand, it greatly exerted the function of nourishing nerves, repairing nerves, and alleviating the pain of the medicine itself. On the other hand, it also stimulates Zusanli acupoints, stimulating its effects of invigorating qi and activating blood, nourishing bones and muscles, resisting pathogens, and so on, which are beneficial to the rehabilitation of ischemic stroke. Although the dosage is small, the acupoints interact, cooperate, and complement each other, and the effect is obvious. Acupoint injection can promote the functional reorganization of the central nervous system of the brain, accelerate the regeneration of tree sprouts and axons, gradually improve the patient's muscle strength, and reduce the degree of spasm and paralysis of the lower limbs [24]. Once the patient's mobility increases, the scope of movement becomes wider, and the living ability naturally improves. The degree of dependence on caregivers will be reduced; self-respect and self-centeredness will be restored and improved accordingly; the quality of life will gradually improve; and the economic and psychological burden will also be reduced. This is consistent with Tang research point of view, both of which are believed to promote lower limb function and activities of daily living and improve the prognostic quality of life [25]. Research data shows that the MBI (lower extremity) scores of patients after the intervention are all higher than before the intervention, and there is a statistical difference (*P* < 0.05); the final score of the experimental group was higher than that of the control group (*P* < 0.05) indicating that it was statistically significant [26]. All show that the intervention measures of acupoint injection are very meaningful and have more advantages [27].

## 5. Conclusion

(1) The method of injecting methylzulanamine at Zusanli acupoint can effectively improve the neurological deficit of patients with ischemic stroke. (2) Injecting methylzulanamine at Zusanli acupoint can effectively improve the motor function of lower limbs in patients with ischemic stroke. (3) The method of injecting methylazuramine at Zusanli acupoint can effectively improve the activities of daily living of patients with ischemic stroke. In the clinical treatment of stroke and its sequelae, although acupoint injection is widely used and has significant effects, there are few studies on the therapeutic effect of a specific single point (Zusanli) on stroke. In terms of medication, methazolamide is mostly used in the treatment of diabetic peripheral neuropathy. This study uses it as a drug to improve the rehabilitation of lower limbs after stroke is also a major breakthrough. The evaluation adopts comprehensive considerations of nerves, sports, and life ability. It is also a bright spot to combine Zusanli acupoint with methylzuanamine (medicine acupoint matching) for the first time to explore the comprehensive effect. Affected by comprehensive factors such as manpower, financial resources, time, and so on, this study only selected 60 patients with ischemic stroke who met the clinical requirements for the study. The sample size was small; only the comparative observation of short-term curative effects was emphasized; and no follow-up treatment was performed. In the future, if conditions permit, multifactor, large sample, and long-term follow-up randomized controlled trials should be considered to provide evidence-based medicine. Most of the evaluation criteria for the curative effect of this project are scale evaluations, which are subjective indicators and lack objective evaluation indicators. Research on laboratory inspections and imaging inspections will be strengthened. In the future, we will seek more scientific, objective, and standardized indicators. This project lacks an objective TCM syndrome differentiation for patients with ischemic stroke. In addition, in acupuncture point injection, the selection of injection points, timing, technique, injection volume, injection course, and stimulus size will be affected by many factors. The size of the impact should also be considered as comprehensive as possible, and it is worthy of our further study.

RETRACTED

## Figures and Tables

**Figure 1:** Acupuncture.

**Figure 2:** Comparison of NIHSS and FMA scores of lower limbs.

**Figure 3:** Comparison of MBI index before/after intervention in group F50, P25, and P75.

**Figure 4:** Comparison of NIHSS and FMA scores of lower limbs in the control group.

**Figure 5:** Comparison of MBI index P50, P25, and P75 before and after intervention.

**Figure 6:** Comparison of NIHSS and FMA scores of lower limbs between two groups.

**Figure 7:** Comparison of MBI Index P50, P25, and P75 between the two groups of patients.

**Table 1:** Comparison of age and course of disease between the two groups.

Project	Test group (*n* = 30)	Control group (*n* = 30)	*t*	*P*
Age	67.67 ± 6.48	68.27 ± 7.08	0.342	0.733
Course of disease (days)	29.27 ± 1.89	29.33 ± 2.89	0.106	0.916

**Table 2:** A comparative example of medication use between the two groups.

Group (*n* = 60)	Antihypertensive drugs (case (%))			Activating blood medicine (case (%))		Antiplatelet aggregation drugs (cases (%))	
	1 type	2 types	3 types	No	Yes	No	Yes
Test group (*n* = 30)	19 (63.3)	8 (26.7)	3 (10.0)	22 (73.3)	8 (26.7)	24 (80.0)	6 (20.0)
Control group (*n* = 30)	21 (70.0)	7 (23.3)	2 (6.7)	20 (66.7)	10 (33.3)	25 (83.3)	5 (16.7)
(*x*^2^/*z*) value	0.579^2^			0.317^1^		0.111^1^	
*P* value	0.562			0.573		0.739	

**Table 3:** Comparison of NIHSS and FMA scores of lower limbs in the two groups.

Project	Test group (*n* = 30)	Control group (*n* = 30)	*t*	*P*
NIHSS score	10.27 ± 1.36	10.2 ± 1.21	0.200	0.842
FMA score	19.47 ± 4.17	19.50 ± 3.99	0.000	1.000

**Table 4:** Comparison of MBI index between the two groups before intervention P50.

Project	Test group (*n* = 30)	Control group (*n* = 30)	*Z*	*P*
MBI index	0 (0, 5)	0 (0, 5)	−0.197	0.844

## Data Availability

The data sets used and analyzed during the current study are available from the corresponding author upon reasonable request.
